The article "{6,6′-Dimeth­oxy-2,2′-[ethane-1,2-diylbis(nitrilo­methyl­idyne)]diphenolato-1κ4 O 1,O 1′,O 6,O 6′:2κ4 O 1,N,N′,O 1′}(ethanol-1κO)-μ-nitrato-1:2κ2 O:O′-dinitrato-1κ4 O,O′-samarium(III)zinc(II)" was retracted in 2010. Reasons: fabricated or falsified data; errors in the data.

# {6,6′-Dimeth­oxy-2,2′-[ethane-1,2-diylbis(nitrilo­methyl­idyne)]diphenolato-1κ^4^ *O* ^1^,*O* ^1′^,*O* ^6^,*O* ^6′^:2κ^4^ *O* ^1^,*N*,*N*′,*O* ^1′^}(ethanol-1κ*O*)-μ-nitrato-1:2κ^2^ *O*:*O*′-dinitrato-1κ^4^ *O*,*O*′-samarium(III)zinc(II)

**DOI:** 10.1107/S1600536809033558

**Published:** 2009-09-05

**Authors:** Qiang Huang, Yu-Hua Sui, Guo-Xiang Zhang

**Affiliations:** a College of Mechanical and Materials Engineering, Jiujiang University, 332005 Jiujiang, JiangXi, People’s Republic of China; b Vacational Education Center of JiLin Oil Feild, 131200 SongYuan, JiLin, People’s Republic of China; c The Pipeline Tools Subsidiary, Well Drilling Technology and Service Corporation of Jilin Oil Field, 131200 SongYuan, JiLin, People’s Republic of China

## Abstract

In the title heteronuclear Zn^II^–Sm^III^ complex, [SmZn(C_18_H_18_N_2_O_4_)(NO_3_)_3_(CH_3_CH_2_OH)], with the hexa­dentate Schiff base compartmental ligand *N*,*N*′-bis­(3-methoxy­salicyl­idene)ethyl­enediamine (H_2_ *L*), the Sm^III^ and Zn^II^ ions are triply bridged by two phenolate O atoms from the Schiff base ligand and one nitrate anion. The five-coordinate Zn^II^ ion is in a square-pyramidal geometry formed by the donor centers of two imine N atoms, two phenolate O atoms and one of the bridging nitrate O atoms. The Sm^III^ center is in a ten-fold coordination of O atoms, involving the phenolate O atoms, two meth­oxy O atoms, one ethanol O atom, and two O atoms from two nitrate anions and one from the bridging nitrate anion. In the crystal, inter­molecular O—H⋯O and C—H⋯O inter­actions generate a layer structure extending parallel to (101).

## Related literature

For the preparation, magnetic and optical properties of 3*d*-4*f* hetorometallic dinuclear complexes, see: Baggio *et al.* (2000 ▶); Caravan *et al.* (1999 ▶); Edder *et al.* (2000 ▶); Knoer *et al.* (2005 ▶).

## Experimental

### 

#### Crystal data

[SmZn(C_18_H_18_N_2_O_4_)(NO_3_)_3_(C_2_H_6_O)]
*M* *_r_* = 774.16
Monoclinic,
*a* = 9.975 (3) Å
*b* = 13.780 (4) Å
*c* = 19.889 (6) Å
β = 91.745 (4)°
*V* = 2732.4 (13) Å^3^
*Z* = 4
Mo *K*α radiation
μ = 3.08 mm^−1^
*T* = 293 K
0.26 × 0.23 × 0.19 mm

#### Data collection

Bruker APEXII area-detector diffractometer
Absorption correction: multi-scan (*SADABS*; Bruker, 2004 ▶) *T*_min_ = 0.501, *T*_max_ = 0.592
16112 measured reflections
4741 independent reflections
4175 reflections with *I* > 2σ(*I*)
*R*_int_ = 0.021

#### Refinement

*R*[*F* ^2^ > 2σ(*F* ^2^)] = 0.027
*wR*(*F* ^2^) = 0.079
*S* = 1.08
4741 reflections
377 parameters
3 restraints
H atoms treated by a mixture of independent and constrained refinement
Δρ_max_ = 0.67 e Å^−3^
Δρ_min_ = −0.70 e Å^−3^

### 

Data collection: *APEX2* (Bruker, 2004 ▶); cell refinement: *SAINT* (Bruker, 2004 ▶); data reduction: *SAINT*; program(s) used to solve structure: *SHELXS97* (Sheldrick, 2008 ▶); program(s) used to refine structure: *SHELXL97* (Sheldrick, 2008 ▶); molecular graphics: *SHELXL97*; software used to prepare material for publication: *SHELXL97* and *publCIF* (Westrip, 2009 ▶).

The article "{6,6′-Dimeth­oxy-2,2′-[ethane-1,2-diylbis(nitrilo­methyl­idyne)]diphenolato-1κ4 O 1,O 1′,O 6,O 6′:2κ4 O 1,N,N′,O 1′}(ethanol-1κO)-μ-nitrato-1:2κ2 O:O′-dinitrato-1κ4 O,O′-samarium(III)zinc(II)" was retracted in 2010. Reasons: fabricated or falsified data; errors in the data.

## Supplementary Material

Crystal structure: contains datablocks I, global. DOI: 10.1107/S1600536809033558/at2862sup1.cif

Structure factors: contains datablocks I. DOI: 10.1107/S1600536809033558/at2862Isup2.hkl

Additional supplementary materials:  crystallographic information; 3D view; checkCIF report

## Figures and Tables

**Table 1:** Hydrogen-bond geometry (Å, °)

*D*—H⋯*A*	*D*—H	H⋯*A*	*D*⋯*A*	*D*—H⋯*A*
C18—H18*B*⋯O9	0.96	2.52	3.237 (6)	132
O14—H14*S*⋯O6^i^	0.855 (19)	1.87 (2)	2.718 (4)	171 (5)
C8—H8⋯O11^ii^	0.93	2.55	3.440 (5)	160

Symmetry codes: (i) ; (ii) .

## supplementary crystallographic information

### Comment

The potential applications of trivalent lanthanide complexes as contrast agent for magnetic resonance imaging and stains for fluorescence imaging have prompted considerable interest in the preparation, magnetic and optical properties of 3 d-4f hetorometallic dinuclear complexes (Baggio *et al.*, 2000; Caravan *et al.*, 1999; Edder *et al.*, 2000; Knoer *et al.*, 2005). we report here the synthesis and X-ray crystal structure analysis of the title complex, (I), a new Zn^II^—Sm^III^ complex with salen-type Schiff base *N*,*N*'-bis(3-methoxysalicylidene) ethylenediamine(H_2_*L*).

Complex (I) crystallizes in the space group *P*2_1_/*n*, with zinc and samarium triply bridged by two phenolate O atoms provided by a salen-type Schiff base ligand and one nitrate. The inner salen-type cavity is occupied by zinc(II), while samarium(III) is present in the open and larger portion of the dinucleating compartmental Schiff base ligand.

The Sm^III^ center has a decacoordination environment of O atoms, involving the phenolate O atoms, two methoxy O atoms, one ethanol O atom, two O atoms from two nitrates and one from the bridging nitrate. The five kinds of Sm—O bond distances are significantly different, the longest being the Sm—*O*(methoxy) separations and the shortest being the Sm—O5(bridging nitrate).

The Zn^II^ is in a square-pyramidal geometry and is five-coordinated by two imine N atoms, two phenolate O atoms and one of the bridging nitrate O atoms.

Adjacent molecules are held together by typical O—H···O hydrogen bonds and weak C—H···O interactions. these link the molecules into a two-dimensional layer structure(Fig 2).

### Experimental

H_2_*L* was prepared by the 2:1 condensation of 3-methoxysalicylaldehyde and ethylenediamine in methanol. Complex (I) was obtained by the treatment of zinc(II) acetate dihydrate (0.188 g, 1 mmol) with H_2_*L*(0.328 g, 1 mmol) in ethanol solution (80 ml) under reflux for 3 h and then for another 3 h after the addition of samarium(III) nitrate hexahydrate(0.444 g, 1 mmol). The reaction mixture was cooled and the resulting precipitate was filtered off, washed with diethyl ether and dried *in vacuo*. Single crystals of (I) suitable for X-ray analysis were obtained by slow evaporation at room temperature of a ethanol solution. Analysis calculated for C_20_H_24_N_5_O_14_SmZn: C 31.03, H 3.12, N 9.05, Sm 19.42, Zn 8.45%; found: C 31.10, H 2.98, N 8.99, Sm 20.01, Zn 8.40%. IR(KBr, cm^-1^): 1640(C=N), 1386,1490(nitrate).

The article "{6,6′-Dimeth­oxy-2,2′-[ethane-1,2-diylbis(nitrilo­methyl­idyne)]diphenolato-1κ4 O 1,O 1′,O 6,O 6′:2κ4 O 1,N,N′,O 1′}(ethanol-1κO)-μ-nitrato-1:2κ2 O:O′-dinitrato-1κ4 O,O′-samarium(III)zinc(II)" was retracted in 2010. Reasons: fabricated or falsified data; errors in the data.

### Refinement

The H atoms were positioned geometrically and treated as riding on their parent atoms, with C—H distances of 0.97 (methylene), 0.96 Å (methyl) and 0.93 Å (aromatic), and with *U*_iso_(H) = 1.5*U*_eq_(C) for methyl H atoms and 1.2*U*_eq_(C) for other H atoms. The hydroxyl H atom, H14s, was located in a difference Fourier map and the O14—H14s was restrained to 0.88 Å.

### Crystal data

**Table:**

[SmZn(C_18_H_18_N_2_O_4_)(NO_3_)_3_(C_2_H_6_O)]	*F*(000) = 1532
*M**_r_* = 774.16	*D*_x_ = 1.882 Mg m^−^^3^
Monoclinic, *P*2_1_/*n*	Mo *K*α radiation, λ = 0.71073 Å
Hall symbol: -P 2yn	Cell parameters from 5725 reflections
*a* = 9.975 (3) Å	θ = 2.5–28.2°
*b* = 13.780 (4) Å	µ = 3.08 mm^−^^1^
*c* = 19.889 (6) Å	*T* = 293 K
β = 91.745 (4)°	Block, yellow
*V* = 2732.4 (13) Å^3^	0.26 × 0.23 × 0.19 mm
*Z* = 4	

### Data collection

**Table:**

Bruker APEXII area-detector diffractometer	4741 independent reflections
Radiation source: fine-focus sealed tube	4175 reflections with *I* > 2σ(*I*)
graphite	*R*_int_ = 0.021
φ and ω scans	θ_max_ = 25.0°, θ_min_ = 1.8°
Absorption correction: multi-scan (*SADABS*; Bruker, 2004)	*h* = −11→11
*T*_min_ = 0.501, *T*_max_ = 0.592	*k* = −15→16
16112 measured reflections	*l* = −23→23

### Refinement

**Table:**

Refinement on *F*^2^	Primary atom site location: structure-invariant direct methods
Least-squares matrix: full	Secondary atom site location: difference Fourier map
*R*[*F*^2^ > 2σ(*F*^2^)] = 0.027	Hydrogen site location: inferred from neighbouring sites
*wR*(*F*^2^) = 0.079	H atoms treated by a mixture of independent and constrained refinement
*S* = 1.08	*w* = 1/[σ^2^(*F*_o_^2^) + (0.045*P*)^2^ + 4.1668*P*] where *P* = (*F*_o_^2^ + 2*F*_c_^2^)/3
4741 reflections	(Δ/σ)_max_ < 0.001
377 parameters	Δρ_max_ = 0.67 e Å^−^^3^
3 restraints	Δρ_min_ = −0.70 e Å^−^^3^

### Special details

**Table:**

Geometry. All e.s.d.'s (except the e.s.d. in the dihedral angle between two l.s. planes) are estimated using the full covariance matrix. The cell e.s.d.'s are taken into account individually in the estimation of e.s.d.'s in distances, angles and torsion angles; correlations between e.s.d.'s in cell parameters are only used when they are defined by crystal symmetry. An approximate (isotropic) treatment of cell e.s.d.'s is used for estimating e.s.d.'s involving l.s. planes.
Refinement. Refinement of *F*^2^ against ALL reflections. The weighted *R*-factor *wR* and goodness of fit *S* are based on *F*^2^, conventional *R*-factors *R* are based on *F*, with *F* set to zero for negative *F*^2^. The threshold expression of *F*^2^ > σ(*F*^2^) is used only for calculating *R*-factors(gt) *etc*. and is not relevant to the choice of reflections for refinement. *R*-factors based on *F*^2^ are statistically about twice as large as those based on *F*, and *R*- factors based on ALL data will be even larger.

The article "{6,6′-Dimeth­oxy-2,2′-[ethane-1,2-diylbis(nitrilo­methyl­idyne)]diphenolato-1κ4 O 1,O 1′,O 6,O 6′:2κ4 O 1,N,N′,O 1′}(ethanol-1κO)-μ-nitrato-1:2κ2 O:O′-dinitrato-1κ4 O,O′-samarium(III)zinc(II)" was retracted in 2010. Reasons: fabricated or falsified data; errors in the data.

### Fractional atomic coordinates and isotropic or equivalent isotropic displacement parameters (Å^2^)

**Table:**

	*x*	*y*	*z*	*U*_iso_*/*U*_eq_	
C1	0.5387 (4)	0.1513 (4)	0.1046 (2)	0.0435 (11)	
H1A	0.6226	0.1846	0.1108	0.065*	
H1B	0.5050	0.1609	0.0594	0.065*	
H1C	0.5517	0.0832	0.1126	0.065*	
C2	0.4878 (4)	0.1904 (3)	0.21745 (19)	0.0287 (8)	
C3	0.4091 (4)	0.2491 (3)	0.25846 (18)	0.0248 (8)	
C4	0.4475 (4)	0.2570 (3)	0.32728 (19)	0.0309 (9)	
C5	0.5626 (4)	0.2059 (3)	0.3513 (2)	0.0405 (11)	
H5	0.5894	0.2119	0.3963	0.049*	
C6	0.6343 (5)	0.1489 (4)	0.3106 (2)	0.0468 (12)	
H6	0.7083	0.1151	0.3280	0.056*	
C7	0.5978 (4)	0.1404 (3)	0.2430 (2)	0.0416 (10)	
H7	0.6473	0.1011	0.2150	0.050*	
C8	0.3727 (4)	0.3097 (3)	0.37649 (19)	0.0325 (9)	
H8	0.4042	0.3070	0.4209	0.039*	
C9	0.1883 (5)	0.4013 (3)	0.4187 (2)	0.0419 (11)	
H9A	0.1913	0.4716	0.4174	0.050*	
H9B	0.2236	0.3797	0.4621	0.050*	
C10	0.0444 (5)	0.3652 (4)	0.4069 (2)	0.0432 (11)	
H10A	0.0380	0.2976	0.4201	0.052*	
H10B	−0.0162	0.4027	0.4340	0.052*	
C11	−0.1155 (4)	0.3718 (3)	0.3160 (2)	0.0376 (10)	
H11	−0.1793	0.3652	0.3488	0.045*	
C12	−0.1630 (4)	0.3768 (3)	0.2471 (2)	0.0337 (9)	
C13	−0.3008 (4)	0.3975 (3)	0.2340 (3)	0.0454 (11)	
H13	−0.3576	0.4041	0.2700	0.054*	
C14	−0.3520 (4)	0.4080 (3)	0.1702 (3)	0.0482 (12)	
H14	−0.4427	0.4212	0.1631	0.058*	
C15	−0.2698 (4)	0.3991 (3)	0.1159 (2)	0.0419 (11)	
H15	−0.3044	0.4081	0.0724	0.050*	
C16	−0.1355 (4)	0.3769 (3)	0.1268 (2)	0.0327 (9)	
C17	−0.0801 (4)	0.3635 (3)	0.1915 (2)	0.0291 (8)	
C18	−0.0918 (5)	0.3868 (4)	0.0095 (2)	0.0523 (13)	
H18A	−0.1594	0.3406	−0.0040	0.078*	
H18B	−0.0188	0.3835	−0.0207	0.078*	
H18C	−0.1295	0.4509	0.0085	0.078*	
C19	0.0334 (4)	0.0595 (3)	0.1448 (3)	0.0453 (11)	
H19A	0.0360	0.0054	0.1761	0.054*	
H19B	0.0421	0.0337	0.0998	0.054*	
C20	−0.0964 (5)	0.1103 (4)	0.1492 (3)	0.0640 (15)	
H20A	−0.1040	0.1376	0.1934	0.096*	
H20B	−0.1683	0.0651	0.1409	0.096*	
H20C	−0.1014	0.1612	0.1163	0.096*	
H14S	0.189 (4)	0.093 (3)	0.1907 (18)	0.045 (14)*	
N1	0.2671 (4)	0.3598 (3)	0.36409 (16)	0.0334 (8)	
N2	0.0069 (4)	0.3757 (3)	0.33567 (17)	0.0365 (8)	
N3	0.2742 (4)	0.5201 (3)	0.18223 (18)	0.0429 (8)	
N4	0.3575 (4)	0.3693 (3)	−0.00107 (19)	0.0461 (10)	
N5	0.1636 (4)	0.1430 (3)	−0.00124 (17)	0.0380 (8)	
O1	0.3020 (3)	0.29131 (19)	0.22943 (13)	0.0285 (6)	
O2	0.0480 (2)	0.3360 (2)	0.19722 (13)	0.0310 (6)	
O3	0.4443 (3)	0.1886 (2)	0.15072 (13)	0.0340 (6)	
O4	−0.0437 (3)	0.3650 (2)	0.07643 (14)	0.0378 (7)	
O5	0.2537 (3)	0.4574 (2)	0.13814 (15)	0.0460 (8)	
O6	0.2370 (3)	0.5111 (2)	0.24316 (13)	0.0334 (6)	
O7	0.3498 (5)	0.6110 (3)	0.1638 (3)	0.0920 (15)	
O8	0.4194 (3)	0.3382 (2)	0.05096 (16)	0.0441 (7)	
O9	0.2306 (3)	0.3687 (2)	−0.00015 (14)	0.0422 (7)	
O10	0.4160 (5)	0.3958 (4)	−0.0499 (2)	0.0997 (17)	
O11	0.0688 (3)	0.1928 (2)	0.02181 (14)	0.0383 (7)	
O12	0.2775 (3)	0.1549 (2)	0.02628 (15)	0.0408 (7)	
O13	0.1458 (4)	0.0871 (3)	−0.04800 (19)	0.0694 (11)	
O14	0.1442 (3)	0.1242 (2)	0.16021 (15)	0.0361 (7)	
Sm1	0.209482 (19)	0.287372 (15)	0.113944 (9)	0.02816 (9)	
Zn1	0.17006 (4)	0.38157 (3)	0.27338 (2)	0.02711 (12)	

The article "{6,6′-Dimeth­oxy-2,2′-[ethane-1,2-diylbis(nitrilo­methyl­idyne)]diphenolato-1κ4 O 1,O 1′,O 6,O 6′:2κ4 O 1,N,N′,O 1′}(ethanol-1κO)-μ-nitrato-1:2κ2 O:O′-dinitrato-1κ4 O,O′-samarium(III)zinc(II)" was retracted in 2010. Reasons: fabricated or falsified data; errors in the data.

### Atomic displacement parameters (Å^2^)

**Table:**

	*U*^11^	*U*^22^	*U*^33^	*U*^12^	*U*^13^	*U*^23^
C1	0.035 (2)	0.060 (3)	0.036 (2)	0.016 (2)	0.0029 (18)	−0.011 (2)
C2	0.0245 (19)	0.034 (2)	0.027 (2)	−0.0018 (16)	−0.0040 (15)	0.0050 (16)
C3	0.0228 (19)	0.028 (2)	0.0233 (19)	−0.0031 (15)	−0.0020 (14)	0.0067 (15)
C4	0.028 (2)	0.038 (2)	0.027 (2)	−0.0031 (17)	−0.0074 (16)	0.0051 (17)
C5	0.035 (2)	0.058 (3)	0.028 (2)	0.001 (2)	−0.0093 (18)	0.0101 (19)
C6	0.036 (2)	0.058 (3)	0.046 (3)	0.012 (2)	−0.012 (2)	0.015 (2)
C7	0.036 (2)	0.045 (3)	0.044 (3)	0.0095 (19)	0.0013 (19)	0.007 (2)
C8	0.036 (2)	0.041 (2)	0.0203 (19)	−0.0063 (18)	−0.0052 (16)	0.0038 (17)
C9	0.056 (3)	0.049 (3)	0.021 (2)	0.003 (2)	0.0044 (18)	−0.0073 (19)
C10	0.052 (3)	0.053 (3)	0.026 (2)	0.004 (2)	0.0140 (19)	−0.0007 (19)
C11	0.035 (2)	0.036 (2)	0.043 (3)	−0.0011 (18)	0.0172 (19)	−0.0053 (19)
C12	0.026 (2)	0.031 (2)	0.045 (2)	−0.0022 (16)	0.0072 (17)	−0.0053 (18)
C13	0.028 (2)	0.041 (3)	0.068 (3)	−0.0012 (19)	0.015 (2)	−0.008 (2)
C14	0.022 (2)	0.049 (3)	0.074 (4)	0.0056 (19)	−0.004 (2)	−0.007 (2)
C15	0.029 (2)	0.038 (3)	0.057 (3)	0.0059 (18)	−0.010 (2)	−0.005 (2)
C16	0.029 (2)	0.027 (2)	0.042 (2)	0.0032 (16)	−0.0028 (17)	−0.0083 (17)
C17	0.025 (2)	0.024 (2)	0.038 (2)	0.0009 (15)	0.0006 (16)	−0.0061 (16)
C18	0.051 (3)	0.066 (3)	0.039 (3)	0.017 (2)	−0.013 (2)	−0.001 (2)
C19	0.038 (3)	0.038 (3)	0.060 (3)	−0.002 (2)	−0.002 (2)	0.006 (2)
C20	0.036 (3)	0.059 (3)	0.097 (5)	−0.002 (2)	0.009 (3)	−0.003 (3)
N1	0.043 (2)	0.0359 (19)	0.0215 (16)	−0.0051 (16)	0.0014 (14)	−0.0033 (14)
N2	0.040 (2)	0.041 (2)	0.0291 (18)	−0.0007 (16)	0.0111 (15)	0.0003 (15)
N3	0.058 (2)	0.038 (2)	0.0329 (14)	0.0040 (17)	0.0048 (15)	−0.0028 (12)
N4	0.053 (3)	0.048 (2)	0.038 (2)	0.0035 (18)	0.0141 (18)	0.0109 (18)
N5	0.047 (2)	0.038 (2)	0.0287 (18)	−0.0019 (17)	−0.0023 (16)	−0.0059 (16)
O1	0.0244 (14)	0.0385 (16)	0.0221 (14)	0.0051 (11)	−0.0042 (10)	−0.0010 (11)
O2	0.0226 (13)	0.0421 (16)	0.0282 (14)	0.0061 (12)	−0.0005 (11)	−0.0067 (12)
O3	0.0251 (14)	0.0489 (17)	0.0279 (15)	0.0091 (12)	−0.0016 (11)	−0.0054 (12)
O4	0.0317 (15)	0.0516 (18)	0.0298 (15)	0.0093 (13)	−0.0054 (12)	−0.0056 (13)
O5	0.071 (2)	0.0360 (17)	0.0308 (15)	−0.0057 (15)	0.0056 (15)	−0.0015 (11)
O6	0.0410 (16)	0.0288 (15)	0.0303 (12)	−0.0026 (12)	0.0015 (11)	−0.0031 (11)
O7	0.114 (4)	0.069 (3)	0.095 (4)	−0.018 (3)	0.033 (3)	−0.002 (2)
O8	0.0332 (16)	0.053 (2)	0.0460 (19)	−0.0035 (14)	−0.0014 (13)	0.0090 (15)
O9	0.0420 (18)	0.054 (2)	0.0309 (16)	0.0052 (14)	−0.0023 (13)	0.0070 (14)
O10	0.085 (3)	0.143 (5)	0.074 (3)	0.015 (3)	0.042 (3)	0.058 (3)
O11	0.0355 (16)	0.0480 (18)	0.0310 (16)	0.0025 (13)	−0.0073 (12)	−0.0040 (13)
O12	0.0341 (17)	0.0488 (19)	0.0393 (17)	0.0041 (13)	−0.0037 (13)	−0.0085 (14)
O13	0.082 (3)	0.069 (3)	0.056 (2)	−0.001 (2)	−0.013 (2)	−0.036 (2)
O14	0.0323 (16)	0.0368 (17)	0.0386 (17)	−0.0058 (12)	−0.0078 (13)	0.0112 (13)
Sm1	0.02985 (13)	0.03342 (14)	0.02110 (13)	0.00080 (8)	−0.00085 (8)	−0.00187 (8)
Zn1	0.0286 (2)	0.0328 (3)	0.0200 (2)	−0.00050 (18)	0.00205 (17)	−0.00135 (17)

The article "{6,6′-Dimeth­oxy-2,2′-[ethane-1,2-diylbis(nitrilo­methyl­idyne)]diphenolato-1κ4 O 1,O 1′,O 6,O 6′:2κ4 O 1,N,N′,O 1′}(ethanol-1κO)-μ-nitrato-1:2κ2 O:O′-dinitrato-1κ4 O,O′-samarium(III)zinc(II)" was retracted in 2010. Reasons: fabricated or falsified data; errors in the data.

### Geometric parameters (Å, °)

**Table:**

C1—O3	1.430 (5)	C17—O2	1.334 (5)
C1—H1A	0.9600	C18—O4	1.433 (5)
C1—H1B	0.9600	C18—H18A	0.9600
C1—H1C	0.9600	C18—H18B	0.9600
C2—C7	1.379 (6)	C18—H18C	0.9600
C2—O3	1.384 (5)	C19—O14	1.446 (5)
C2—C3	1.406 (6)	C19—C20	1.477 (7)
C3—O1	1.333 (4)	C19—H19A	0.9700
C3—C4	1.414 (5)	C19—H19B	0.9700
C4—C5	1.418 (6)	C20—H20A	0.9600
C4—C8	1.444 (6)	C20—H20B	0.9600
C5—C6	1.348 (7)	C20—H20C	0.9600
C5—H5	0.9300	N1—Zn1	2.043 (3)
C6—C7	1.387 (6)	N2—Zn1	2.077 (3)
C6—H6	0.9300	N3—O5	1.244 (5)
C7—H7	0.9300	N3—O6	1.284 (4)
C8—N1	1.277 (5)	N3—O7	1.512 (6)
C8—H8	0.9300	N4—O10	1.205 (5)
C9—N1	1.474 (5)	N4—O8	1.264 (5)
C9—C10	1.530 (7)	N4—O9	1.267 (5)
C9—H9A	0.9700	N5—O13	1.217 (5)
C9—H9B	0.9700	N5—O12	1.257 (4)
C10—N2	1.462 (5)	N5—O11	1.265 (5)
C10—H10A	0.9700	O1—Zn1	2.028 (3)
C10—H10B	0.9700	O1—Sm1	2.450 (3)
C11—N2	1.272 (6)	O2—Zn1	2.014 (3)
C11—C12	1.438 (6)	O2—Sm1	2.439 (3)
C11—H11	0.9300	O3—Sm1	2.787 (3)
C12—C17	1.413 (6)	O4—Sm1	2.822 (3)
C12—C13	1.420 (6)	O5—Sm1	2.429 (3)
C13—C14	1.362 (7)	O6—Zn1	2.004 (3)
C13—H13	0.9300	O8—Sm1	2.570 (3)
C14—C15	1.380 (7)	O9—Sm1	2.545 (3)
C14—H14	0.9300	O11—Sm1	2.621 (3)
C15—C16	1.385 (6)	O12—Sm1	2.627 (3)
C15—H15	0.9300	O14—Sm1	2.523 (3)
C16—O4	1.387 (5)	O14—H14S	0.855 (19)
C16—C17	1.398 (6)		
			
O3—C1—H1A	109.5	O5—N3—O7	118.5 (4)
O3—C1—H1B	109.5	O6—N3—O7	118.0 (3)
H1A—C1—H1B	109.5	O10—N4—O8	121.8 (4)
O3—C1—H1C	109.5	O10—N4—O9	121.5 (4)
H1A—C1—H1C	109.5	O8—N4—O9	116.7 (3)
H1B—C1—H1C	109.5	O13—N5—O12	121.7 (4)
C7—C2—O3	124.6 (4)	O13—N5—O11	121.8 (4)
C7—C2—C3	121.7 (4)	O12—N5—O11	116.6 (3)
O3—C2—C3	113.7 (3)	C3—O1—Zn1	127.1 (2)
O1—C3—C2	117.0 (3)	C3—O1—Sm1	132.1 (2)
O1—C3—C4	125.1 (3)	Zn1—O1—Sm1	100.77 (10)
C2—C3—C4	117.8 (3)	C17—O2—Zn1	122.1 (2)
C3—C4—C5	118.7 (4)	C17—O2—Sm1	132.1 (2)
C3—C4—C8	124.4 (4)	Zn1—O2—Sm1	101.52 (10)
C5—C4—C8	116.8 (4)	C2—O3—C1	115.4 (3)
C6—C5—C4	121.8 (4)	C2—O3—Sm1	118.7 (2)
C6—C5—H5	119.1	C1—O3—Sm1	124.9 (2)
C4—C5—H5	119.1	C16—O4—C18	115.8 (3)
C5—C6—C7	120.1 (4)	C16—O4—Sm1	117.3 (2)
C5—C6—H6	119.9	C18—O4—Sm1	126.7 (3)
C7—C6—H6	119.9	N3—O5—Sm1	146.6 (3)
C2—C7—C6	119.9 (4)	N3—O6—Zn1	118.6 (2)
C2—C7—H7	120.1	N4—O8—Sm1	96.1 (2)
C6—C7—H7	120.1	N4—O9—Sm1	97.2 (2)
N1—C8—C4	125.5 (4)	N5—O11—Sm1	97.6 (2)
N1—C8—H8	117.3	N5—O12—Sm1	97.6 (2)
C4—C8—H8	117.3	C19—O14—Sm1	132.6 (2)
N1—C9—C10	106.2 (3)	C19—O14—H14S	103 (3)
N1—C9—H9A	110.5	Sm1—O14—H14S	125 (3)
C10—C9—H9A	110.5	O5—Sm1—O2	73.74 (10)
N1—C9—H9B	110.5	O5—Sm1—O1	74.45 (10)
C10—C9—H9B	110.5	O2—Sm1—O1	66.10 (9)
H9A—C9—H9B	108.7	O5—Sm1—O14	146.58 (10)
N2—C10—C9	109.1 (3)	O2—Sm1—O14	79.28 (10)
N2—C10—H10A	109.9	O1—Sm1—O14	76.81 (9)
C9—C10—H10A	109.9	O5—Sm1—O9	74.48 (10)
N2—C10—H10B	109.9	O2—Sm1—O9	123.96 (10)
C9—C10—H10B	109.9	O1—Sm1—O9	141.92 (10)
H10A—C10—H10B	108.3	O14—Sm1—O9	138.33 (10)
N2—C11—C12	125.3 (4)	O5—Sm1—O8	71.83 (11)
N2—C11—H11	117.4	O2—Sm1—O8	145.17 (10)
C12—C11—H11	117.4	O1—Sm1—O8	99.31 (9)
C17—C12—C13	118.0 (4)	O14—Sm1—O8	130.09 (10)
C17—C12—C11	123.7 (4)	O9—Sm1—O8	49.82 (10)
C13—C12—C11	118.2 (4)	O5—Sm1—O11	135.09 (10)
C14—C13—C12	121.6 (4)	O2—Sm1—O11	105.13 (9)
C14—C13—H13	119.2	O1—Sm1—O11	147.66 (9)
C12—C13—H13	119.2	O14—Sm1—O11	70.91 (9)
C13—C14—C15	120.4 (4)	O9—Sm1—O11	69.69 (10)
C13—C14—H14	119.8	O8—Sm1—O11	102.80 (10)
C15—C14—H14	119.8	O5—Sm1—O12	138.80 (10)
C14—C15—C16	119.5 (4)	O2—Sm1—O12	146.17 (9)
C14—C15—H15	120.3	O1—Sm1—O12	122.69 (9)
C16—C15—H15	120.3	O14—Sm1—O12	72.40 (10)
C15—C16—O4	124.8 (4)	O9—Sm1—O12	71.60 (10)
C15—C16—C17	121.8 (4)	O8—Sm1—O12	68.60 (10)
O4—C16—C17	113.5 (3)	O11—Sm1—O12	48.25 (9)
O2—C17—C16	117.8 (3)	O5—Sm1—O3	105.83 (10)
O2—C17—C12	123.5 (4)	O2—Sm1—O3	121.53 (8)
C16—C17—C12	118.6 (4)	O1—Sm1—O3	58.34 (8)
O4—C18—H18A	109.5	O14—Sm1—O3	72.15 (9)
O4—C18—H18B	109.5	O9—Sm1—O3	110.93 (9)
H18A—C18—H18B	109.5	O8—Sm1—O3	64.54 (9)
O4—C18—H18C	109.5	O11—Sm1—O3	111.62 (9)
H18A—C18—H18C	109.5	O12—Sm1—O3	66.62 (8)
H18B—C18—H18C	109.5	O5—Sm1—O4	80.93 (10)
O14—C19—C20	111.1 (4)	O2—Sm1—O4	58.08 (8)
O14—C19—H19A	109.4	O1—Sm1—O4	123.23 (8)
C20—C19—H19A	109.4	O14—Sm1—O4	101.26 (9)
O14—C19—H19B	109.4	O9—Sm1—O4	72.24 (9)
C20—C19—H19B	109.4	O8—Sm1—O4	120.25 (9)
H19A—C19—H19B	108.0	O11—Sm1—O4	63.13 (9)
C19—C20—H20A	109.5	O12—Sm1—O4	109.57 (9)
C19—C20—H20B	109.5	O3—Sm1—O4	173.01 (9)
H20A—C20—H20B	109.5	O6—Zn1—O2	104.55 (12)
C19—C20—H20C	109.5	O6—Zn1—O1	100.96 (11)
H20A—C20—H20C	109.5	O2—Zn1—O1	82.54 (10)
H20B—C20—H20C	109.5	O6—Zn1—N1	104.02 (13)
C8—N1—C9	121.5 (3)	O2—Zn1—N1	151.32 (13)
C8—N1—Zn1	128.0 (3)	O1—Zn1—N1	89.69 (12)
C9—N1—Zn1	110.2 (3)	O6—Zn1—N2	119.22 (13)
C11—N2—C10	120.6 (4)	O2—Zn1—N2	88.27 (13)
C11—N2—Zn1	125.5 (3)	O1—Zn1—N2	139.80 (13)
C10—N2—Zn1	113.6 (3)	N1—Zn1—N2	79.99 (14)
O5—N3—O6	123.4 (4)		

The article "{6,6′-Dimeth­oxy-2,2′-[ethane-1,2-diylbis(nitrilo­methyl­idyne)]diphenolato-1κ4 O 1,O 1′,O 6,O 6′:2κ4 O 1,N,N′,O 1′}(ethanol-1κO)-μ-nitrato-1:2κ2 O:O′-dinitrato-1κ4 O,O′-samarium(III)zinc(II)" was retracted in 2010. Reasons: fabricated or falsified data; errors in the data.

### Hydrogen-bond geometry (Å, °)

**Table:**

*D*—H···*A*	*D*—H	H···*A*	*D*···*A*	*D*—H···*A*
C1—H1B···O12	0.96	2.35	2.995 (5)	125
C18—H18B···O9	0.96	2.52	3.237 (6)	132
O14—H14S···O6^i^	0.86 (2)	1.87 (2)	2.718 (4)	171 (5)
C8—H8···O11^ii^	0.93	2.55	3.440 (5)	160

Symmetry codes: (i) −*x*+1/2, *y*−1/2, −*z*+1/2; (ii) *x*+1/2, −*y*+1/2, *z*+1/2.
